The article "Comparison of CNN Algorithms for Feature Extraction on Fundus Images to Detect Glaucoma" was published in 2022. Journal: J Healthc Eng.

# Comparison of CNN Algorithms for Feature Extraction on Fundus Images to Detect Glaucoma

**DOI:** 10.1155/2022/7873300

**Published:** 2022-01-07

**Authors:** V. Sunanthini, J. Deny, E. Govinda Kumar, S. Vairaprakash, Petchinathan Govindan, S. Sudha, V. Muneeswaran, M. Thilagaraj

**Affiliations:** ^1^Department of Electronics and Instrumentation Engineering, Easwari Engineering College, Chennai, India; ^2^Department of Electronics and Communication Engineering, Kalasalingam Academy of Research and Education, Srivilliputhur, India; ^3^Department of Electronics and Instrumentation Engineering, Karpagam College of Engineering, Coimbatore, India; ^4^Department of Electronics and Communication Engineering, Ramco Institute of Technology, Rajapalayam, India; ^5^Department of Electrical and Electronics Technology, Ethiopian Technical University, Addis Ababa, Ethiopia

## Abstract

Glaucoma is a disease where the optic nerve of the eyes is smashed up due to the building up of pressure inside the vision point. This has no symptoms at the initial stages, and hence, patients with this disease cannot identify them at the beginning stage. It is explained as if the pressure in the eye increases, then it will hurt the optic nerve which sends images to the brain. This will lead to permanent vision loss or total blindness. The existing method used for the detection of glaucoma includes k-nearest neighbour and support vector machine algorithms. The k-nearest neighbour algorithm and support vector machine algorithm are the machine learning methods for both categorization and degeneration problems. The drawback in using these algorithms is that we can get accuracy level only up to 80%. The proposed methods in this study focus on the convolution neural network for the recognition of glaucoma. In this study, 2 architectures of VGG, Inception method, AlexNet, GoogLeNet, and ResNet architectures which provide accuracy levels up to 100% are presented.

## 1. Introduction

A persistent vision problem which destructs the optic nerve of the eye is called glaucoma. Every year, a number of people are getting affected by this invisible disease. The problem is not known at the initial stages. Only when the vision starts to narrow down, a person will be able to identify. It is due to the excess fluid which builds up in some portion of the eye. This added fluid raises the pressure in the eye which deteriorates the optic nerve. The excess fluid secreted in the eye is drained out through the drainage angle, thereby keeping the pressure of the eye stable for a normal person. For the person affected with glaucoma, the excess water is not rained out properly, thereby increasing the pressure of the eye [1]. The symptoms of this disease differ according to the type and the stage of our condition. Open angle glaucoma has a symptom of patchy spots in one or both the eyes. Closed angle glaucoma has the symptoms of blurred vision and headache. Glaucoma as shown in Figure 1 is diagnosed by various tests such as measuring the intraocular pressure, testing the optic nerve damage, measuring the corneal thickness, investigating the contour and nature of the visual part, verifying the entire field of vision, testing the position in the eye where the iris and cornea gather, and observing the drainage viewpoint and also cup to disc ratio [2]. The existing clinical methods are expensive and require experienced clinicians to use them.

## 2. Proposed Framework

Fundus images have been used for detecting glaucoma and diabetic retinopathy [3]. The damage caused to optic nerve fibre is detected using the features of fundus images [4]. The drawback seen in the above methods is that glaucoma cannot be diagnosed at an earlier stage. To overcome these problems, the image processing methods are used to achieve more precise output. CNN architectures used in this system are VGG16 [5], VGG19, Inception, AlexNet, GoogLeNet method, and ResNet method. Feature extractions like training process rate, iteration, confusion matrix, specificity, sensitivity, and accuracy represented in the numerical and graphical method are also used. Training images and validation images are the input images that undergo processing. Under training images, the images of both glaucoma and the healthy person are given. Validation image consists of a predefined image with normal parameters to be compared with glaucoma image. All the images fed in the training image will be compared with the preset validation image for detection of glaucoma. Then, the glaucoma detected images will reach the preprocessing stage. From there, these images will pass into various architectures like VGG16, VGG19, Inception, Exception method, GoogLeNet method, and SqueezeNet method. Then, it will pass into layer preparation. The more the number of layers, the more will be the accuracy level for glaucoma detection [6]. Then, it undergoes data training for producing results. Then, the results obtained will be in the form of confusion matrix, specificity, sensitivity, and accuracy.

## 3. Design Modules

### 3.1. VGG16 Architecture

VGG16 is an extensively used neural network architecture. Accuracy found in VGG16 is up to 92.2%, equipped with a dataset of million images. The large kernel-sized filters with multiple kernels one after another are built in this model. VGG16 is trained with large time consumption. This architecture has structure size of 244 ∗ 244. In a preprocessing step, the average RGB value is deducted from each pixel in an image as shown in Figure 2. When the initial step is finished, the images are stepped to a pile of density layers with tiny opened field filters in the dimensions of (3 × 3). In some programs, the filter size is set to (1 × 1), which can be recognized as alteration of the input channels [7–9].

Many convolution layers are there in VGG16, whereas these layers are followed by 5 grouping layers which in turn is carried by spatial pooling. Among the 5 max pooling layers, first layer and second layer have 4096 ways each, and the third layer has 1000-part divisions. The last layer has the SoftMax layer. These 5 max pooling layers are carried by spatial grouping. The hidden layers of VGG16 as shown in Figure 3 are followed by activation function. There is a fully connected layer configuration which always remains the same.

Images from the ImageNet dataset are used for training the data by VGG19 as this network is in CNN architecture. The images can be categorized by making use of this network to get all object classifications This network has deep layers and can also be recognized and identified using the algorithms. The rich feature representations for a wide range of images can be learnt by this network. This architecture has an image input size of 224 × 224, as shown in Figure 4. The new set of images can be classified using this network for more trained networks in Matlab. A fixed size of RGB image is given as input to this network where the matrix has the shape (224 × 224 × 3).

The kernels of (3 × 3) with a step size of 1 pixel are preprocessed, and the average RGB value is deducted from each pixel, calculated on the training set. It helps them to envelop the entire perception of the illustration. Spatial filling is made to maintain the spatial precision of the image. This is proceeded by rectified linear unit (ReLu) to add nonlinearity and to make the model categorization better and to increase the calculation time as the prior models used or sigmoid tasks, and they are confirmed with improved results. The completely joined layers can be computed from which first and second layers are of size 4096, third layer with 1000 channels for 1000-way categorization and the last layer is for a SoftMax task.

### 3.2. AlexNet Architecture

AlexNet architecture consists of 8 layers. There are 5 convolution layers and 3 totally linked layers. The 2 structures are made to overlap grouping connections to remove a minimum feature. All the fully connected layers and output of the layers can be connected to the linear activation kernels. The key proportions of the AlexNet structure is 256 × 256 × 3. It means that the input to the network consists of RGB which has 3 channels and image of 256 × 256 pixels, respectively, as shown in Figure 5. This structure is with 6,50,000 neurons and 60 million parameters. In order to cut the extra fitting during the components working process, drop out layers are used by networks. In the forward pass and back propagation, the neurons which are crashed off cannot be added and participated. A stochastic slope optimization role with momentum, batch size, and weight decomposed set to 0.9, 128, and 0.0005 correspondingly are used by this model. A learning rate of 0.001 is used equally by all the layers. Both dropout layers and data augmentation for over fitting during training are used. AlexNet consists of 8 *l* channels with weights: the first 5 are convolution and the remaining 3 are wholly linked up. The output of the final fully linked layer is fed to a 1000-way SoftMax. It develops a distribution over the 1000 class labels. The system boosts the multinomial logistic degeneration point. The network can be linked to maximize the mean across training cases of the likelihood of the correct label under expected allotment [10, 11].

### 3.3. GoogLeNet

GoogLeNet is based on the activations which are either unnecessary (zero) or redundant. Hence, the architecture of a deep network is a sparse connection between the activations, so that all 512 input channels have not a connection with all the 512 output channels. To prune out such connections which would result in a sparse weight/connection, some techniques can be used. To remove the fully connected layers with good accuracy, a large network width and depth is used. It achieves 93.3% accuracy, and it is much faster than VGG architectures. The evaluation of accuracy of GoogLeNet is harder to do, and it requires more human work to increase an accuracy, and an error rate of 6% was achieved by GoogLeNet in previous studies. It is subjected to training the experts who can develop the accuracy percentage up to 3–5%, respectively, as shown in Figure 6. The CNN network is used and implemented in a novel element which is dubbed an inception module. This layer uses image distortion and normalization. The 22-layer deep CNN and reduced parameter rate from 60 to 4 million are constructed. In order to reduce the parameters rate gradually, this structure is based on convolutions [12].

### 3.4. ResNet

Deep learning is the method of learning hierarchical set of representations, and its low mid and high-level features are learnt. In images, it is analogous of learning edges, shapes, and then objects. More layers have to enhance the levels of the features and previous models. The ResNet typically have depth of 16 and 30 layers. This shows how ResNet is better than other architectures. If a shallow architecture is considered to its deeper counterpart, the entrenched model would just need to clone the thinner model with character mappings. It is learnt that a deeper model should produce no higher preparation error than its thinner complement. It found how to make the figure significantly deeper than like the VGG19 layers, but with this mechanism, the 1600 layers do not present properly. It is proposed in this thesis that it is due to proper behavior. The picture is resized with its tinier side arbitrarily tested in 224,580 for scale extension. A 256 × 256 yield is arbitrarily tested from an illustration or its straight spin, with the per-pixel average minimized. The studying rate begins from 0.01 and is divided by 10 when the error plateaus and the models are trained up to 600 × 100000 iterations, as shown in Figure 7. A weight decay of 0.00001 is used and a momentum is 0.09 [13, 14].

### 3.5. Inception ResNet V2

In image recognition performances, deep convolution networks brought advances in recent years. Inception architecture can be given as an example as it shows the performance at relatively low computational cost. It is identified that traditional architecture with a residual connection in conjunction has given state of the art evaluation. The performance of Inception V2 is similar to that of the performance of the Inception V3 network. The empirical evidence show that residual connections initiate the inception networks training. The improved expensive inception can be implemented by a slight margin without remaining associations. Some restructured designs for remaining inception networks can be executed. The distinct edge identification accomplishment on the categorization job is improved significantly by the assigned network. The established ranging alleviates the extensive and outstanding inception networks and is demonstrated and shown in Figure 8. An accuracy of 3.08% is realized on sample set of the ImageNet categorization. Inception ResNet V2 is a convolution neural network. From the ImageNet database, this network is prepared on more than a millions of sample data from the record of ImageNet. This network is classified into object divisions such as mouse and modem. Enhanced features for a broad collection of images are realized by the complex system [15].

### 3.6. Future Scope

The image processing methods are extensively used for automatic identification of optic disc, blood vessels, and analysis of texture. The examination of these CNNs and tested results are proven to be an important analysis to the glaucoma categorization study using fundus images. The above computational methods can be used to resolve the obstacle of this crisis. The model has been developed to distinguish diseased and nondiseased eyes using the CNN algorithm. In forthcoming work, the additional parameters such as retinal rim width, retinal area, horizontal cup-disc ratio, and rim-to-disc ratio can also be computed to show the evolution of growth. They will play a vital task in the medical field and present various methods for the identification of the glaucoma in early stages.

## 4. Result

The accuracy as shown in Figure 9 of the computed data processing networks is good. The first layer of the spare self-encoder and the training result are used as the next layer. The sensitivity is shown in Figure 10. The preset instruction parameter can be set from the result. The trained output makes the layer by layer to obtain a deep learning model. The characteristics depth representation is obtained, and the classifier is added. The loss function for the trained and finely tuned model is built and assembled. After the algorithm is tested, the comparison of provisional diagnosis is established. It can be examined by the ophthalmologist with the results of the planned method. Hence, it is concluded that the proposed method achieves increased accuracy. In a ROC curve, the accuracy is plotted in the function of the special cutoff points of constraints. The region under the ROC curve is the evaluation of a factor which can distinguish between two investigative groups, and the ROC curves are shown in Figures 11–17. The novelty of this work is that we have compared various architectures for this glaucoma characterizing and presented the results with best accuracy for the database that we have considered.

## 5. Conclusion

The presence of the disc is a strong indicator of glaucoma disease. In the convolution neural network, the various ImageNet-learnt CNN structures (VGG16, VGG19, Inception V2, and ResNet50) were analyzed and used as a glaucoma disease classifier. The inception structure illustrates greatest accomplishment for glaucoma taxonomy which is the swapping between AUC and the amount of constraints of the CNN. In the existing system, KNN and SVM architectures were used. In this work, the database has composed of 2450 normal images and 853 glaucomatous images and for further comparison. Based on 1706 images, an average AUC of 0.9605 with 92% interval of 96.92–98.07%, an average specificity of 0.8580, and an average sensitivity of 0.9346 were achieved. It is summarized that the identification of glaucoma with the morphological appearances were obtained more precisely by applying CNN operated algorithms.

## Figures and Tables

**Figure 1:** Glaucoma.

**Figure 2:** Confusion matrix: VGG16.

**Figure 3:** VGG16-layer preparation.

**Figure 4:** Confusion matrix: VGG19.

**Figure 5:** Confusion matrix, AlexNet.

**Figure 6:** Confusion matrix, GoogLeNet.

**Figure 7:** Confusion matrix, ResNet.

**Figure 8:** Confusion matrix, Inception ResNet V2.

**Figure 9:** Accuracy graph.

**Figure 10:** Sensitivity graph.

**Figure 11:** ROC curve, VGG16.

**Figure 12:** ROC curve, VGG19.

**Figure 13:** ROC curve, GoogLeNet.

**Figure 14:** ROC curve, AlexNet.

**Figure 15:** ROC curve, Inception.

**Figure 16:** ROC curve, ResNet50.

**Figure 17:** ROC curve, ResNet101.

## Data Availability

The data used to support the findings of this study are available from the corresponding author upon request.
